# Determination of multidrug resistance mechanisms in *Clostridium perfringens* type A isolates using RNA sequencing and 2D-electrophoresis

**DOI:** 10.1590/1414-431X20187044

**Published:** 2018-06-11

**Authors:** Yu-Hua Ma, Gui-Sheng Ye

**Affiliations:** 1 State Key Laboratory of Plateau Ecology and Agriculture, Qinghai University, Xining, China; 2 College of Agriculture and Animal Husbandry, Qinghai University, Xining, China

**Keywords:** Clostridium perfringens, Multidrug resistance, RNA sequencing, 2D-electrophoresis, Molecular mechanism

## Abstract

In this study, we screened differentially expressed genes in a multidrug-resistant isolate strain of *Clostridium perfringens* by RNA sequencing. We also separated and identified differentially expressed proteins (DEPs) in the isolate strain by two-dimensional electrophoresis (2-DE) and mass spectrometry (MS). The RNA sequencing results showed that, compared with the control strain, 1128 genes were differentially expressed in the isolate strain, and these included 227 up-regulated genes and 901 down-regulated genes. Bioinformatics analysis identified the following genes and gene categories that are potentially involved in multidrug resistance (MDR) in the isolate strain: drug transport, drug response, hydrolase activity, transmembrane transporter, transferase activity, amidase transmembrane transporter, efflux transmembrane transporter, bacterial chemotaxis, ABC transporter, and others. The results of the 2-DE showed that 70 proteins were differentially expressed in the isolate strain, 45 of which were up-regulated and 25 down-regulated. Twenty-seven DEPs were identified by MS and these included the following protein categories: ribosome, antimicrobial peptide resistance, and ABC transporter, all of which may be involved in MDR in the isolate strain of C. perfringens. The results provide reference data for further investigations on the drug resistant molecular mechanisms of C. perfringens.

## Introduction

*Clostridium perfringens*, an important zoonotic pathogen, is capable of causing necrotic enteritis and food poisoning in humans (1,2). Bacterial drug resistance can occur through inherent gene mutations and foreign gene acquisition (3). With inherent gene mutation acquisition, the resistance gene exists in the bacterial genome, and the drug resistance is typically species-specific, such as penicillin resistance in *Pneumococcus* (4). When bacteria develop drug resistance through the acquisition of foreign genes, the resistance gene may be located in the bacterial genome, or in a plasmid, transposon, or integron; hence, resistance genes can be spread via plasmids, transposons and integrons among the various carriers, making bacterial drug-resistance patterns more complex and diverse. The inactivating or modifying enzymes produced by bacteria mainly cause a loss of biological activity in an antibiotic, and this loss involves bacterial β-lactam-inactivating enzymes, aminoglycoside-modifying enzymes, and chloramphenicol acetyltransferases (5).

Under antibiotic pressure, an alteration of the target bacterial protein can occur in the drug-binding site of the intracellular membrane and this reduces the affinity of the drug for its target, thereby eliminating the efficacy of the antibiotic. This is a common mechanism of drug resistance in bacteria (6). The efflux pump is another primary cause of bacteria resistance to many drugs (7), such as ATP-binding cassette, ABC transporter, and drug-resistant nodulation division family (8). Due to the efflux pump, *Escherichia coli*, *Staphylococcus aureus*, etc. have multiple resistance to tetracycline, fluoroquinolones, and β-lactam among others (9).

The *C. perfringens* TetA(P) protein is an endometrial protein that regulates tetracycline active efflux. It consists of 420 amino acids and 12 transmembrane domains (10). The resistance mode by reducing membrane permeability is relatively rare in gram-positive bacteria, but vancomycin-resistant *Staphylococcus aureus* can specifically modify the cell wall to reduce permeability, thereby reducing the amount of drug entering the cell (11). *Streptococcus pneumoniae* can produce *VncR-VncS* and other cell wall regulators to change the cell wall permeability and develop resistance (12).

Bacterial biofilm is an important cause of bacterial resistance (13); it can reduce the penetration of antibacterials due to the barrier function of extracellular polysaccharides (14). The growth of bacteria in biofilm is slow and the sensitivity to antibiotics is reduced (15). The induced expression of *rpoS* gene in the biofilm formation stage of *Escherichia coli* may be caused by the formation of drug-resistant subgroups in the deep layer of the mature biofilm (16). *C. perfringens* can form biofilms, and type IV *pilus* and *CcpA* protein are necessary for biofilm formation. The biofilm from *C. perfringens* resists oxygen and antibiotics effectively (17).

In this study, we analyzed differentially expressed genes (DEGs) and differentially expressed proteins (DEPs) in a multidrug resistance (MDR) isolate of type A *C. perfringens*. The study used RNA sequencing (RNA-Seq), two-dimensional electrophoresis (2-DE), and mass spectrometry (MS) to investigate the transcriptome and proteome of the MDR isolate and a control strain of C. perfringens.

## Material and Methods

### Strains

An MDR strain of *C. perfringens* type A was isolated, identified, and preserved by the Laboratory of Animal Disease based at the Qinghai-Tibet Plateau in the Department of Veterinary Medicine, College of Agriculture and Animal Husbandry, Qinghai University, China (18). The standard *C. perfringens* type A strain, CICC22949, purchased from the China Center of Industrial Culture Collection, was used as the control strain. In the preliminary experiments on the isolate strain of *C. perfringens*, we found that the minimum inhibitory concentrations of kanamycin sulfate, minocycline hydrochloride, clindamycin hydrochloride, doxycycline hydrochloride, and novobiocin were higher than those of the control strain.

### Total RNA extraction, cDNA library construction, and sequencing

*C. perfringens* were grown overnight at 37°C in liquid medium of sulfate glycolate after sterilization. The cells were harvested by centrifugation at 10,625 *g* for 3 min at room temperature when *C. perfringens* were grown with an initial OD600 of 0.6. Total RNA of the *C. perfringens* isolate strain and control strain were extracted using the RNA Isolater total RNA extraction reagent (Cat#401, Vazyme, China) according the manufacturer's instructions. An RNA integrity number was determined using an Agilent 2100 bioanalyzer (Agilent Technologies, USA). After quantification, 10 µg of the extracted RNA was digested by DNase I at 37°C for 30 min. Ribosomal RNA was removed using a Ribo-Zero™ magnetic kit (Epicentre, USA). The cDNA library was constructed using the NEB Next¯ UltraTM directional RNA library prep kit from Illumina (NEB, USA). Random primers and first strand synthesis reaction buffer (NEB) were added to the mRNA solution to allow cDNA synthesis to occur. Following purification, end repair and joint connection were conducted to give 300–500 bp ligated cDNA molecules. After polymerase chain reaction (PCR) amplification and library construction, sequencing was performed using Illumina Hiseq™ 2500.

### Genome comparison and DEG analysis

The raw sequencing reads were filtered for quality control to obtain clean reads. These reads were then mapped to the reference genome using SOAP2 (19). The distribution and coverage of the reads on the reference sequence were analyzed. DEGs were screened by analysis of the significance of digital gene expression profiles (20), followed by enrichment analysis of gene ontology (GO) terms by GO TermFinder software (http://smd.stanford.edu/help/GO-TermFinder/GO_TermFinder_help.shtml) and KEGG pathways (21).

### Two-dimensional electrophoresis

Culture sample (1 g) was decanted and 1 mL of lysis buffer (9 mol/L UREA, 4% CHAPS, 1% IPG buffer, 1% DTT was added. The sample was disrupted by ultrasonication (80–100 W, 3 min) and centrifuged (10,625 *g* for 30 min at 4°C) to remove the precipitate. Next, 1 mL of pre-cooled acetone was added and the sample was kept at −20°C overnight. The supernatant was removed after centrifugation (10,625 *g* for 30 min at 4°C). The precipitate was dried and 500 μL of protein hydration solution was added. The extracted protein was quantified and used for 2-DE. Briefly, 150 µg of the protein sample was removed, dry strips were prepared (pH 3–10 NL IPG), and run for the first-dimension isoelectric focusing. The equilibrated strips were placed in the gel slab for the second-dimensional sodium dodecyl sulfate-polyacrylamide gel electrophoresis. After electrophoresis, the gel was stained with Coomassie blue. Following decolorization, the gel was scanned by ImageScanner (GE Healthcare, USA).

### MS detection and DEP analysis

Selected granules were excised from the gel and transferred to 1.5-mL tubes for decolorization. The sample was digested with trypsin and 100 µL of 60% acetonitrile (ACN); 0.1% trifluoroacetic acid (TFA) was added. The mixture was ultrasonicated for 15 min and then lyophilized. After lyophilization, 2 mL of the digested sample was collected and 20% ACN was added. A 1-mL aliquot of the sample was spotted onto the sample target and 0.5 μL of supersaturated CHA solution was spotted onto the corresponding target. The sample was air dried and the sample target was blown with nitrogen gas before being placed into the target slot for the MS analysis. The laser source was Nd:YAG laser with 355 nm wavelength, and the peptide mass fingerprinting mass scan range was 800–4000 Da. Parent ions with signal-to-noise ratios greater than 50 were selected for tandem MS (MS/MS) analysis. The MS/MS was performed with a laser excitation of 2500 times and 2 kV of collision energy, and with the collision-induced decomposition shut down. The MS data were analyzed using Mascot (SCIEX, USA). GO and Kyoto Encyclopedia of Genes and Genomes (KEGG) analyses (http://www.kegg.jp/) of the DEPs were conducted.

## Results

### Transcriptome sequencing data and DEG analysis

A total of 28,563,164 reads were obtained from the MDR isolate strain of *C. perfringens* by transcriptome sequencing. Specifically, 83.97% of the reads were mapped to the *C. perfringens* genome, 60.71% were mapped to *C. perfringens* genes, and the unique matches reached 83.35%. Concurrently, 26,254,552 reads were obtained from the *C. perfringens* control strain by transcriptome sequencing. Specifically, 89.41% of the reads were mapped to the *C. perfringens* genome, 72.6% mapped to *C. perfringens* genes, and the unique matches reached 88.65%.

For the MDR isolate strain of *C. perfringens*, the vast majority of gene coverages were higher than 10%; this included 2000 gene coverages between 90 and 100%. For the control strain, all gene coverages were higher than 10%; this included 2437 gene coverages between 90 and 100%.

A total of 1128 DEGs (FDR≤0.05 and |log2Ratio|≥1), including 227 up-regulated genes and 901 down-regulated genes, were screened in the MDR isolate strain relative to the control strain (Figure 1).

**Figure 1.** Differentially expressed genes (DEGs) in the multidrug resistance (MDR) isolate strain of *C. perfringens.* The red color represents up-regulated tags, the green color represents down-regulated tags (fold change) and the blue color represents no significant DEGs. FDR: false discovery rate.

We performed GO and KEGG enrichment analyses on 1128 DEGs in the MDR isolate strain of *C. perfringens*. The results showed that these DEGs participated in 648 biological processes (Figure S1A) wherein defense responses, drug transport, drug responses, and lactamase transport may be related to multidrug resistance in the MDR isolate strain of *C. perfringens*. These DEGs are derived from 80 cellular components (Figure S1B) wherein the ABC transporter, ATP-dependent transmembrane transporter, transmembrane transporter, protein membrane complex, and ribosome may be related to multidrug resistance in the MDR isolate strain of *C. perfringens*. Moreover, these DEGs have 399 molecular functions (Figure S1B) wherein hydrolase, transport protein, transmembrane transporter activity, transferase activity, amidase transmembrane transporter, transcription factor activity, and efflux transmembrane transporter activity may be related to multidrug resistance in the MDR isolate strain of *C. perfringens*.

The 1128 DEGs are involved in 122 KEGG pathways (Figure 2) wherein bacterial chemotaxis, ABC transporter, and β-lactam resistance may be associated with multidrug resistance in the MDR isolate strain of *C. perfringens*.

**Figure 2.** KEGG enrichment pathway of differentially expressed genes (DEGs) in the multidrug resistance isolate strain of *C. perfringens*. The top 20 enriched pathways are shown in the graph, different color means different Q-value, and the size of the bubble represents the number of DEGs.

### 2-DE, MS, and DEP analyses

The 2-DE results (Figure 3) showed clear protein spots for the MDR isolate strain of *C. perfringens* and the control strain. The trend of the proteins was consistent within each group, with good reproducibility. Next, an image analysis was conducted using ImageScanner and PDquest 8.0 (Bio-Rad, USA) software, and the DEPs were screened using the following criteria: fold changes >2 or <0.5 for the analytical values, and P-values <0.05 by the *t*-test. A total of 70 DEPs, 45 of which were up-regulated and 25 were down-regulated, were identified in the isolate strain relative to the control strain.

**Figure 3.** Comparative analysis of proteins of *C. perfringens* by 2D- electrophoresis. The image shows the differential expression of protein spots from the proteins extracted from (*left*) multidrug resistance isolate strain of *C. perfringens*, and (*right*) control strain. Proteins whose fold change were higher than 2 or less than 0.5 were selected for further analysis. The arrows refer to the differentially expressed protein spots.

Twenty-seven DEP spots with large fold-changes for up-regulated expression were selected from the MDR isolate strain of *C. perfringens* for enzymatic hydrolysis and desalination in the gel. The digested samples were re-dissolved with ACN and spotted onto the sample target for Maldi-TOF/TOF analysis. The MS data were used for protein identification using Mascot search software. The results showed that the 27 protein spots were identified successfully.

GO and KEGG enrichment analyses were performed on the amino acid sequences of the 27 DEP spots successfully identified by MS. The results showed that the DEPs found in the MDR isolate strain of *C. perfringens* participated in 292 biological processes (Figure S2A), 111 of which were significantly enriched. These DEPs were related to 44 cellular components (Figure S2B), 18 of which were significantly enriched. Moreover, these DEPs were involved in 142 molecular functions (Figure S2C), 37 of which were significantly enriched.

The 27 DEPs participating in 24 KEGG pathways (Figure 4) include ribosomes, antibiotic biosynthesis, antimicrobial peptide resistance, and ABC transporters. The ribosomal pathway, antimicrobial peptide resistance, and ABC transporters may be related to multidrug resistance in the MDR isolate strain of *C. perfringens*.

**Figure 4.** KEGG pathway enrichment analysis of differentially expressed proteins in the multidrug resistance isolate strain of *C. perfringens*. Differentially expressed proteins were categorized according to their gene ontology terms and in each category the number of proteins and their P-values are shown in the graph. The X-axis shows the percentage of differentially enriched proteins.

## Discussion

Bacteria will trigger a variety of mechanisms against drugs under the sustained pressure of antibiotics. β-lactamase is a primary cause of resistance to β-lactam antibiotics (22); its encoding gene can spread among bacteria by transformation, transduction, conjugation, and other ways, such as in ESBLs-producing bacteria (23). Aminoglycoside modifying enzymes can help bacteria to develop resistance to aminoglycoside antibiotics (24), as the encoding gene can transfer among bacteria through plasmid conjugation, and cause drug resistance (25). Bacteria can also develop drug resistance by increasing the number of target proteins (26). Resistance to β-lactam antibiotics can be caused by changing the number of penicillin binding proteins or deleting it. This kind of drug resistance is common in bacteria, which is dependent on β-lactam antibiotics rather than β-lactamases (27). The resistance of the bacteria to rifampin is due to the change in the beta subunit of the RNA polymerase in the bacteria, thus reducing the drug's binding capacity and developing resistance (28).

*C. perfringens* isolated from piglets in Thailand was reported to have an MDR phenotype (29). This bacterium has also been reported to be capable of inactivating antibiotics via production of drug-inactivating or drug-modifying enzymes (30). In chloramphenicol-resistant *C. perfringens*, the product encoded by the catP resistance gene, which is located on the Tn4453 transposon, can inactivate chloramphenicol and spread via plasmid conjugation (31). In lincomycin-resistant *C. perfringens*, the transposon-located tlSCpe8 nucleotidyltransferase, which is encoded by the *tInuP* resistance gene and spreads by plasmid conjugation, can inactivate lincomycin (32). Additionally, because of gene transfer, tet(M) resistance gene appeared in *C. perfringens* type C, carrying tetB resistance gene (33). *C. perfringens* can develop quinolone resistance by altering the sites of drug action in the genes encoding DNA gyrase and topoisomerase IV. Mutated gryA DNA gyrasegenein *C. perfringens*, and the mutant bacterium grown in an environment with gatifloxacin and ciprofloxacin showed a certain degree of resistance to these antibiotics (34). Additionally, *C. perfringens* acquired linezolid resistance via a new mutation in the highly conserved region of the 50S ribosomal protein L4 gene, rplD (35). When a drug reaches a certain concentration in bacteria, the expression of proteins related to the active efflux system increases, thereby pumping the drug out of the cells. By transferring a putative coding gene of an ABC transporter from a ciprofloxacin-resistant *C. perfringens* strain into a wild-type strain, a study found that not only was the accumulation of ethidium bromide reduced in the recombinant strain, but also the accumulation of norfloxacin and ciprofloxacin was reduced in the cells (36).

In this study, we screened 1128 DEGs from a MDR isolate strain of *C. perfringens* using RNA-Seq. Bioinformatics analysis showed that these genes participated in biological pathways including drug transport, drug response, amidase transport, hydrolase activity, transferase activity, along with an amidase transmembrane transporter, efflux transmembrane transporter, bacterial chemotaxis, ABC transporters, and a β-lactam resistance gene, all of which may be related to multidrug resistance in the isolate strain of *C. perfringens* type A. Furthermore, we obtained 70 DEP spots, including 45 that were up-regulated and 25 that were down-regulated in the MDR isolate strain of *C. perfringens* by 2-DE. Of these, 27 protein spots with relatively large fold-changes in up-regulated expression were identified by MS, and these proteins participate in various biological pathways. The proteins in these spots, which are potentially related to multidrug resistance in the MDR isolate strain of *C. perfringens*, include ribosomes, antimicrobial peptide resistance determinants, and ABC transporters.

## Supplementary Material

Click here to view [pdf]
